# Circular RNA_HIPK3-Targeting miR-93-5p Regulates KLF9 Expression Level to Control Acute Kidney Injury

**DOI:** 10.1155/2023/1318817

**Published:** 2023-02-16

**Authors:** Zha Zhengbiao, Chen Liang, Zheng Zhi, Pan Youmin

**Affiliations:** ^1^Department of Cardiovascular Surgery, Tongji Hospital, Tongji Medical College, Huazhong University of Science and Technology, China; ^2^Department of Infection, Tongji Hospital, Tongji Medical College, Huazhong University of Science and Technology, China

## Abstract

Acute kidney injury (AKI) is a clinical syndrome caused by various reasons that results in the rapid decline of renal function in a short period of time. Severe AKI can lead to multiple organ dysfunction syndrome. Circular RNA HIPK3 (circHIPK3) derived from the *HIPK3* gene is involved in multiple inflammatory processes. The present research was performed to explore the function of circHIPK3 on AKI. The AKI model was established by ischemia/reperfusion (I/R) in C57BL/6 mice or hypoxia/reoxygenation (H/R) in HK-2 cells. The function and mechanism of circHIPK3 on AKI were explored via biochemical index measurement; hematoxylin and eosin (HE) staining; 3-(4,5-dimethylthiazol-2-yl)-2,5-diphenyltetrazolium bromide (MTT); flow cytometry; enzyme-linked immunosorbent assay (ELISA); western blot; quantitative real-time polymerase chain reaction (RT-qPCR); detection of reactive oxygen species (ROS) and adenosine triphosphate (ATP); and luciferase reporter assays. circHIPK3 was upregulated in kidney tissues of I/R-induced mice and in H/R-treated HK-2 cells, while the microRNA- (miR-) 93-5p level was decreased in H/R-stimulated HK-2 cells. Furthermore, circHIPK3 silencing or miR-93-5p overexpression could reduce the level of proinflammatory factors and oxidative stress and recover the cell viability in H/R-stimulated HK-2 cells. Meanwhile, the luciferase assay showed that Krüppel-like transcription factor 9 (KLF9) was the downstream target of miR-93-5p. Forced expression of KLF9 blocked the function of miR-93-5p on H/R-treated HK-2 cells. Knockdown of circHIPK3 improved the renal function and reduced the apoptosis level *in vivo*. In conclusion, circHIPK3 knockdown alleviated oxidative stress and apoptosis and inhibited inflammation in AKI via miR-93-5p-mediated downregulation of the KLF9 signal pathway.

## 1. Introduction

Renal ischemia/reperfusion injury is an important factor leading to acute kidney injury (AKI), delayed recovery of transplanted renal function, and even acute renal failure in severe cases [1, 2]. In the process of renal ischemia, endothelial cells are damaged to induce the production of endothelin, the expression of various receptors, the oxygen-free radical production, and Ca^2+^ overload. These various factors together cause renal microcirculation disorder and hemodynamic changes. In the process of renal reperfusion, cellular structure destruction and metabolic disorders are more serious than these during ischemia, and renal tubular epithelial cells located in the medulla trigger inflammatory responses and lead to cell edema [3–5]. At present, due to the unclear pathogenesis of renal ischemia/reperfusion, there is no specific treatment to reduce its incidence and improve its cure rate. Therefore, understanding the molecular pathogenesis of renal ischemia/reperfusion injury can effectively contribute to the progression, identify the preventive treatment, and block the incidence of renal ischemia/reperfusion injury.

Plenty of researches show that circRNA is involved in the biological processes such as mRNA splicing and transcription and RNA degradation and translation and is closely related to the occurrence and development of a variety of human diseases such as cancers, nervous system disorders, and cardiovascular diseases [6, 7]. Functionally, circRNAs have competitive binding sites for miRNA, which can regulate miRNA activity and ultimately affect the expression of downstream target genes of miRNA [8]. circRNAs participate in the regulation of organ ischemia/reperfusion injury. For instance, circVMA21 inhibits apoptosis and inflammation in sepsis-associated AKI models through the miR-9-3p/SMG1 axis [9]. circ_0114427 can regulate ATF3 by sponging miR-494 to be involved in AKI [10]. Forced expression of circYAP1 reduces inflammation and ROS production in ischemia/reperfusion-treated cells by sponging to miR-21-5p [11]. These findings suggest that circRNAs are new molecular targets for precision diagnosis and treatment of ischemia/reperfusion diseases. circHIPK3 (has_circRNA_000284) is produced from exon2 of the HIPK3 gene and the most abundant spliceosome in the circRNAs of the HIPK3 gene [12]. circHIPK3 has been demonstrated to be dysregulated in various diseases, such as cancers [13, 14], diabetes [15], and fibrosis [13–19]. More importantly, circHIPK3 can sponge diverse miRNAs to regulate the diseases progression. circHIPK3 sponges miR-382-5p to regulate DUSP1 to alleviate neuronal apoptosis and inflammatory response in spinal cord injury [20]. circHIPK3 modulates cell proliferation and migration through the miR-124/AKT3 axis in esophageal squamous cell carcinoma [14]. However, the role of circHIPK3 in renal ischemia/reperfusion injury is still unknown.

Here, we found that circHIPK3 was upregulated in AKI. Silencing of circHIPK3 reduced oxidative stress, apoptosis, and inflammation in both the mouse model and HK-2 cells. Furthermore, we identified miR-95-3p as the direct target of circHIPK3, and Krüppel-like transcription factor 9 (KLF9) would be a downstream protein of the circHIPK3/miR-95-3p axis. In summary, we found that circHIPK3 knockdown could alleviate renal AKI via regulating the miR-95-3p/KLF9 signaling pathway.

## 2. Materials and Methods

### 2.1. Animals

C57BL/6 mice (6-8 weeks, ~25 g, male) were purchased from Charles River (Beijing, China) and kept at the animal center for more than one week before the following experimental procedures. All experimental mice were fed at 22°C in standard breeding cages with a standard condition. The Laboratory Animal Ethics Committee of Tongji Hospital approved all experimental procedures using the C57BL/6 mice.

### 2.2. AKI Model Establishment

Mice were subjected to acute ischemia and reperfusion (I/R) treatment to induce ischemic renal AKI as in a previous report [21]. Mice were anesthetized with 50 mg/kg (body weight) pentobarbital sodium. After deep anesthesia, the back of the mouse was opened with a 1-5 cm long incision, and both renal pedicles were clipped with a micro noninvasive hemostatic clamp for 25 min and then treated with reperfusion for 6 h. Mice in the sham group received the same operation without clamping of kidney pedicles. After the operation, the backs were sutured and the mice were put back into the cage for recovery. In addition, to explore the role of circHIPK3 in vivo, adenovirus vector plasmids including AAV9-si-circHIPK3 and AAV9-si-negative control (AAV9-si-NC) were bought from GenePharma (Shanghai, China) and injected into mice by tail vein 21 days before I/R surgery. Mice were intraperitoneally injected with pentobarbital sodium and were euthanatized via excessive anesthesia with a dose of 250 mg/kg [22]. Their blood and kidney tissues were harvested and processed for biochemical, pathological, and immunoblotting analyses.

### 2.3. Biochemical Index Measurement

After reperfusion, about 2 mL of blood samples was gathered from each mouse via the posterior orbital venous plexus. The blood samples were then centrifuged at 4,000 × *g* for 15 min, and the serum samples were collected and used for the determination of urea nitrogen (BUN), uric acid (UA), and creatinine abundance (CREA) using a Roche Cobas C111 analyzer (Roche, Switzerland). At least three biological repeats were performed for statistical comparisons of BUN, UA, and CREA between different groups.

### 2.4. Hematoxylin and Eosin (H&E) Staining

Kidney tissues were isolated and stained with H&E (G1120, Solarbio, Beijing, China). The tissues were fixed in 4% paraformaldehyde (P1110, Solarbio) for 1 day and embedded in paraffin (YA0012, Solarbio). The tissue was sectioned about 4 *μ*m. The slices were stained with hematoxylin, eosin, and toluidine blue and then were used to observe the pathological changes of the tissues under a light microscope (BX43, Olympus, Tokyo, Japan).

### 2.5. Cell Culture

The human renal proximal tubular epithelial cell line (HK-2) was incubated at 37°C in 10% FBS (SH30413.03, Hyclone, South America) contained DMEM (SH30285.FS, Hyclone) in 5% CO_2_ and 95% air. The cell hypoxia/reoxygenation (H/R) model was established as in a previous report [23]. Briefly, HK-2 cells were exposed to hypoxia 1% oxygen, 94% nitrogen, and 5% CO_2_ for 6 h in DMEM. Subsequently, the culture plates were placed in a normal cell incubator (5% CO_2_ and 95% air) for reoxygenation for 6 h.

### 2.6. 3-(4,5-Dimethylthiazol-2-yl)-2,5-diphenyltetrazolium Bromide (MTT) Assay

HK-2 cells with an inoculation density of 1 × 10^5^ cells/well were sowed into 96-well plates and incubated at 37°C in 5% CO_2_ for 24 h. After cells were incubated with 10 *μ*L of MTT solution (C0009S, Beyotime, Shanghai, China) for 4 h, the culture supernatant was removed, and each well was appended with 100 *μ*L of DMSO to dissolve the crystals. The absorbance at 570 nm was detected using the microplate reader (Tecan, Switzerland).

### 2.7. Flow Cytometry

HK-2 cells were plated into 24-well plates at a density of 2.5 × 10^5^ cells/well and cultured at 37°C in 5% CO_2_ overnight. Then, cells were gathered, washed with phosphate buffer saline (PBS) (C0221A, Beyotime), resuspended with 0.5 mL of bind buffer, and stained with 5 *μ*L of propidium iodide (PI) (P1304MP, Thermo Fisher Scientific, Waltham, MA, USA) and 5 *μ*L of Annexin V/FITC (BMS306FI-100, Thermo Fisher Scientific) at room temperature for 15 min. The cell apoptosis was determined on a FACScan flow cytometer using CellQuest software (BD Biosciences, NJ, USA).

### 2.8. Enzyme-Linked Immunosorbent Assay (ELISA)

The concentrations of interleukin- (IL-) 1*β*, IL-6, and tumor necrosis factor- (TNF-) *α* in HK-2 cells were detected via the Human IL-1*β* ELISA Kit (PI305, Beyotime), Human IL-6 ELISA Kit (PI330, Beyotime), and Human TNF-*α* ELISA Kit (PT518, Beyotime), respectively. The concentrations of IL-1*β*, IL-6, and TNF-*α* in kidney tissues were measured via the Mouse IL-1*β* ELISA Kit (PI301, Beyotime), Mouse IL-6 ELISA Kit (PI326, Beyotime), and Mouse TNF-*α* ELISA Kit (PT512, Beyotime), respectively.

### 2.9. Western Blot

The protein levels were assessed via western blotting. The protein samples from HK-2 cells and kidney tissues were lysed with the RIPA lysis buffer (P0013B, Beyotime), and the protein concentration was determined via the BCA kit (P0012S, Beyotime, China). 50-60 *μ*g of protein samples was separated via sodium dodecyl sulfate-polyacrylamide gel electrophoresis (SDS-PAGE) on a 12% gel and transferred to nitrocellulose membranes (HF18002S25, Merck, NJ, USA). The blot was then incubated in a blocking solution (5% defatted dry milk (P0216, Beyotime)), dissolved in a phosphate buffer saline buffer (PBS, C0221A, Beyotime) followed by washes with PBS, and incubated overnight in PBS containing antibodies (anti-Bcl2 (12789-1-AP, Proteintech, Wuhan, China), anti-Bax (50599-2-Ig, Proteintech), anti-Cytochrome c (Cyt-c) (66264-1-Ig, Proteintech), anti-KLF9 (ab227920, Abcam, Cambridge, UK), and anti-GAPDH (10494-1-AP, Proteintech)) diluted to 1 : 500. The blots were then washed with PBST (PBS containing Tween 20 (ST825, Beyotime)) and incubated for 1 h in PBS containing peroxidase-conjugated anti-mouse/rabbit IgG (PR30009, Proteintech) diluted to 1 : 8000. The blot was developed with the chemiluminescence ECL kit (PE0010, Solarbio, Beijing, China) using the Omega Lum W Chemiluminescence Imaging System (Aplegen, USA), and the optical density was measured using the Image Studio Software. The results were normalized via the loading control (GAPDH).

### 2.10. Quantitative Real-Time Polymerase Chain Reaction

Total RNAs from HK-2 cells and kidney tissues were collected via the TRIzol solution (15596026, Invitrogen, CA, USA). 500 ng of RNA was reverse transcribed into cDNA using the HiScript II Q RT SuperMix (R223-01, Vazyme, Nanjing, China). Quantitative real-time PCR was performed in an ABI 7500 Fast System using the qPCR SYBR Green Master Mix (4309155, Thermo Fisher, MA, USA). The PCR amplification conditions were 94°C for 10 min, 94°C for 10 s, and 60°C for 45 s for 40 cycles. *GAPDH* acted as the internal reference. The expressions of genes were calculated with the comparative threshold cycle method (2^-△△CT^ method), in which ΔΔCT = ΔCT_treatment_ − ΔCT_control_ and ΔCT = Ct_target_ − Ct_reference_. The primers are shown in Table 1.

### 2.11. Reactive Oxygen Species (ROS) Production Detection

The Cellular ROS Assay Kit (ab186027) was purchased from Abcam. Cells were cultured and collected at 10^4^ cells/100 *μ*L per well. Furthermore, 100 *μ*L/well of ROS Red Working Solution was added into the cell plate and incubated in a 37°C/5% CO_2_ incubator for 1 h. Fluorescence activity was measured at Ex/Em = 520/605 nm (cut-off 590 nm) with the bottom read mode. The final results were normalized by the control group.

### 2.12. ATP Measurement Assay

The ATP Assay Kit (S0026, Beyotime, China) was employed to measure the cellular ATP content. Briefly, HK-2 cells were seeded in 12-well plates. After treatment, the cells were lysed with buffer and centrifuged at 12000 × *g* for 5 min at 4°C. The supernatant was collected. Luminance was measured via a monochromator microplate reader (Tecan). The data were normalized by the control group.

### 2.13. Luciferase Reporter Assay

The binding sites between circHIPK3 and miR-93-5p, as well as these between miR-93-5p and KLF9, were predicated by the starBase databases (https://starbase.sysu.edu.cn/starbase2/index.php). HEK293 cells were transfected with 20 mmol/L of miR-93-5p mimic or miR-NC (GenePharma) together with circHIPK3-WT/circHIPK3-mutation or KLF9-WT/KLF9-mutation. Luciferase activity was determined with the Dual Luciferase Reporter Assay Kit (E1910, Promega, Beijing, China) on GloMax 20/20 (Promega) at 48 h after the transfection.

### 2.14. Statistical Analysis

All data were analyzed as the mean ± SD. Statistical significances were measured via the paired Student's *t*-test between two groups and the one-way analysis of variance (ANOVA) for more than two groups followed by the post hoc Bonferroni test using the SPSS 26.0 software (IBM, Armonk, New York, USA). *P* < 0.05 was regarded as a significant difference.

## 3. Results

### 3.1. circHIPK3 Was Upregulated *In Vivo* and *In Vitro*

circHIPK3 plays an important role in I/R injury which occurs in a variety of organs [24–27]. To investigate the abnormal gene expression of *circHIPK3* in response to renal AKI, mice were subjected to renal I/R. Comparing with the sham group, the serum levels of CREA, BUN, and UA were significantly upregulated in the I/R group (Figure 1(a)). Then, the kidney was removed and H&E staining was performed, and tubular dilatation and necrosis were observed in the I/R group (Figure 1(b)). The serum levels of inflammatory cytokines IL-1*β*, IL-6, and TNF-*α* were upregulated in the I/R group (Figure 1(c)). The decreased expression of Bcl2 and increased expression of Bax and Cytochrome c (Cyt-c) were discovered, suggesting the inducing apoptosis in the I/R group (Figure 1(d)). The upregulation of circHIPK3 was found in the I/R group compared with the sham group (Figure 1(e)). In addition, HK-2 cells underwent hypoxia/reoxygenation (H/R) or control treatment. Compared with the control group, the levels of IL-1*β*, IL-6, and TNF-*α* were markedly upregulated in H/R-treated HK-2 cells (Figure 1(f)). The increased apoptosis level was assessed by detecting the expression of Bcl2, Bax, and Cyt-c (Figure 1(g)). The MTT assay showed the decreased cell viability in H/R-treated HK-2 cells compared with the control group (Figure 1(h)). Meanwhile, H/R induced the increased production of ROS (Figure 1(i)) and decreased level of ATP (Figure 1(j)). Consistent with *in vivo* results, the circHIPK3 level was elevated after H/R (Figure 1(k)). These results suggested that the expression of circHIPK3 was upregulated in I/R-treated mice and in H/R-treated HK-2 cells.

### 3.2. Silencing of circHIPK3 Could Alleviate the AKI *In Vitro*

To explore the function of circHIPK3, si-circHIPK3 and si-circRNA NC were transfected into HK-2 cells. All three si-circHIPK3 inhibited the expression of circHIPK3, among which si-circHIPK3#1 displayed the best interference efficiency (Figure 2(a)). Thus, si-circHIPK3#1 was used in the following experiments. Silencing of circHIPK3 improved cell viability in H/R-treated HK-2 cells (Figure 2(b)). si-circHIPK3#1 prevented the increased level of inflammatory cytokines in HK-2 cells induced by H/R treatment (Figure 2(c)). Besides, knockdown of circHIPK3 could significantly reduce the protein expression of Bax and Cyt-c with enhanced expression of the Bcl2 protein in H/R-treated HK-2 cells (Figure 2(d)). circHIPK3 downregulation reversed ROS generation (Figure 2(e)) and recovered the ATP content in H/R-treated HK-2 cells (Figure 2(f)). In summary, knockdown of circHIPK3 improved the AKI in HK-2 cells.

### 3.3. circHIPK3 Interacting with miR-93-5p Participated in AKI

Emerging researches have shown that circRNAs can function as miRNA sponges to regulate downstream targets [28]. Bioinformatics starBase databases predicted that there were binding sites between circHIPK3 and miR-93-5p (Figure 3(a)). To verify the targeting relationship between circHIPK3 and miR-93-5p, mutant circHIPK3 and wild-type circHIPK3 were constructed. Then, we performed luciferase reporter assay in HEK293 cells. As shown in Figure 3(a), the decreased luciferase activity was observed in cotransfection with WT-circHIPK3 and the miR-93-5p mimic, suggesting a direct bind between circHIPK3 and miR-93-5p. Additionally, the level of miR-93-5p was downregulated both *in vivo* and *in vitro* (Figures 3(b) and 3(c)). circHIPK3 overexpression plasmid and miR-93-5p mimic were cotransfected into HK-2 cells. The circHIPK3 and miR-93-5p level was detected via qRT-PCR (Figure 3(d)). Forced expression of circHIPK3 further aggravated H/R-induced cell viability (Figure 3(e)), inflammatory cytokine level (Figure 3(f)), ROS level (Figure 3(g)), and ATP content (Figure 3(h)), and the miR-93-5p mimic could block the effect of the circHIPK3 plasmid on these indexes (Figures 3(e)–3(h)). Flow cytometry results also showed that the apoptosis rate was further induced by circHIPK3 which was blocked by the miR-93-5p mimic (Figure 3(i)). The above results showed that circHIPK3 could act as a sponge for miR-93-5p in I/R-stimulated HK-2 cells.

### 3.4. miR-93-5p Binding with KLF9 Regulated Kidney Injury *In Vitro*

Next, we forecasted that KLF9 may be a target of miR-93-5p, which was verified via the luciferase assay (Figure 4(a)). Meanwhile, the mRNA level of KLF9 was upregulated both *in vivo* and *in vitro* (Figures 4(b) and 4(c)). Western blot assay exhibited the similar results (Figures 4(d) and 4(e)). We added miR-93-5p mimics and the KLF9 vector into HK-2 cells and found that KLF9 recovered the level of miR-93-5p and KLF9 (Figure 4(f)). miR-93-5p mimics showed the similar function with si-circHIPK3 on cell viability, ROS level, ATP content, and apoptosis rate in H/R-treated HK-2 cells, while overexpression of KLF9 inhibited the favorable effect of miR-93-5p mimics on H/R-treated HK-2 cells (Figures 4(g)–4(j)). Taken together, KLF9 might be a target gene for miR-93-5p.

### 3.5. circHIPK3 Regulated AKI by Mediating miR-93-5p/KLF9 Axis *In Vivo*

To verify our results, we constructed the adenovirus vector plasmid, AAV9-si-circHIPK3/AAV9-si-negative control (AAV9-si-NC). The mice were injected with AAV9-si-NC or AAV9-si-circHIPK3 21 days before I/R surgery by tail vein. After operation, the kidneys in all groups were collected, and the levels of circHIPK3, miR-93-5p, and KLF9 were detected. circHIPK3 injection induced the upregulation of circHIPK3 and KLF9 and inhibited the expression of miR-93-5p (Figure 5(a)). The serum levels of CREA, BUN, and UA were significantly upregulated in the I/R group, which was recovered by si-circHIPK3 infection (Figure 5(b)). AAV9-si-circHIPK3 injection mice showed improved tubular dilatation and necrosis compared with the AAV9-si-NC group after I/R (Figure 5(c)). Knockdown of circHIPK3 inhibited I/R-induced apoptosis in vivo, which was indicated by TUNEL staining and western blot assay (Figures 5(d) and 5(f)). AAV9-si-circHIPK3 injection decreased the levels of proinflammatory factors in the I/R group (Figure 5(e)). Together, silencing of circHIPK3 could alleviate AKI via the miR-93-5p/KLF9 signal pathway.

## 4. Discussion

When severe ischemia reperfusion injury occurs in the kidney, it will not only cause glomerular injury and renal failure but also cause chronic renal tubulointerstitial fibrosis [29, 30]. With the long-term development of fibrosis, renal injury caused by ischemia reperfusion can turn into chronic kidney disease, even the end of life. Appropriate animal models can simulate the dynamic changes in the development of the disease and may reveal the molecular regulatory mechanisms in patients [3, 4, 31]. Here, we demonstrated that circHIPK3 was involved in renal AKI by controlling apoptosis, oxidative stress, and inflammation via the miR-93-5p/KLF9 axis.

The role of circRNAs in disease has received increasing attention. Although the role of circRNAs in certain kidney diseases has been reported, such as lupus nephritis and hypertensive nephropathy [32, 33], their function in renal AKI is unclear. circHIPK3 plays an important role in the physiological and pathological processes of multiple organs, especially organ ischemia/reperfusion injury. Wu et al. [34] demonstrated that circHIPK3 was abnormally elevated in the myocardial infarction mouse heart. Interference the circHIPK3 expression could reduce infarction size and apoptosis. The author also revealed that circHIPK3 could regulate the Rac1/PI3K/AKT signal pathway by sponging miR-93-5p. Cheng et al. [35] showed that circHIPK3 could control AKT3 via sponging miR-29b in myocardial ischemia/reperfusion injury. Furthermore, Qiu et al. [25] disclosed that circHIPK3 could promote autophagy and apoptosis in H/R-induced cardiomyocytes by regulating ATF7 via sponging miR-20-5b. Our data showed that circHIPK3 was upregulated in I/R- and H/R-induced renal AKI. Silencing of circHIPK3 could inhibit apoptosis, oxidative stress, and inflammation *in vivo* and *in vitro*, and circHIPK3 knockdown also downregulated the ROS level and recovered the ATP content. These data suggested that circHIPK3 contributed to the oxidation stress, inflammation, and apoptosis during I/R-induced AKI *in vivo* and *in vitro*.

In previous research, miR-93-5p participated in AKI progression by regulating the downstream target. circ-FANCA controlled LPS-induced cell injury by sponging miR-93-5p. Furthermore, miR-93-5p overexpression inhibited LPS-treated HK-2 cell injury by targeting OXSR1. circ-FANCA triggered OXSR1 expression by binding with miR-93-5p [36]. miR-93-5p was also a downstream target of lncRNA NEAT1, and inhibition of NEAT1 blocked LPS-induced damage by inducing miR-93-5p expression in HK-2 cells [37]. Juan et al. [38] also exhibited that exosome-miR-93-5p is involved in sepsis-induced AKI via the influence of pyroptosis in renal epithelial cells. Here, the bioinformatics website predicted that miR-93-5p could interact with circHIPK3. The luciferase assay showed that circHIPK3 could bind with miR-93-5p. The miR-93-5p mimic blocked the proapoptosis and inflammation of circHIPK3 on HK-2 cells, which suggested that miR-93-5p was a downstream target of circHIPK3.

KLF9 is a transcription factor that regulates oxidative stress. It is involved in a wide range of neural development, cell differentiation, proliferation, and apoptosis [39–41]. As a target of miR-218-5p, KLF9 controlled the autophagy, apoptosis, and oxidative stress by regulating the JAK2/STAT3 signaling pathway in rheumatoid arthritis synovial fibroblasts [39]. Furthermore, KLF9 induced mitochondrial dysfunction and ROS accumulation in high glucose-induced SH-SY5Y cells via bupivacaine neurotoxicity [42]. Yan et al. [40] also demonstrated that KLF9 could sharpen the oxidative stress and ROS level in ischemia injury in cardiomyocytes. In our research, we found that KLF9 was a downstream target of miR-93-5p, which was involved in circHIPK3-regulating AKI progression.

## 5. Conclusion

Our research indicated that the circHIPK3 was upregulated in I/R-induced mice and H/R-treated HK-2 cells. Silencing of circHIPK3 improved cell apoptosis, oxidative stress, and inflammation in H/R-treated HK-2 cells. Furthermore, circHIPK3 initiated the reduction of miR-93-5p expression and sponged to miR-93-5p. miR-93-5p overexpression could block the injury induced by circHIPK3 in I/R-treated HK-2 cells. As the downstream target of miR-93-5p, KLF9 was involved in circHIPK3/miR-93-5p-regulating AKI progression. At present, we have exposed the function of circHIPK3 knockdown *in vivo*. To further explore and verify the downstream signal pathway, we gained or lost the function of miR-93-5p and KLF9 *in vivo*. Furthermore, we would collect the plasma of clinical renal failure patients to analyze the potential of circHIPK3 as a biomarker in AKI, which provided an underlying diagnosis and treatment target for AKI.

## Figures and Tables

**Figure 1:** circHIPK3 is upregulated in acute kidney injury. (a) The level of serum CREA, BUN, and uric acid in I/R and sham groups. (b) Representative H&E images are shown in I/R and sham groups. (c) The level of IL-1*β*, IL-6, and TNF-*α* was detected via ELISA. (d) The level of apoptosis-associated protein (Bcl2, Bax, and Cyt-c) was measured via western blot. (e) The level of circHIPK3 was assessed in the I/R and sham groups. (f) H/R treatment was performed in the HK-2 cell, and the level of IL-1*β*, IL-6, and TNF-*α* was detected via ELISA. (g) The level of apoptosis-associated protein was measured via western blot. (h). Cell viability was detected via MTT. (i) The production of ROS was evaluated via the Reactive Oxygen Species Assay Kit. (j) The content of ATP was measured via the ATP Assay Kit. (k) The level of circHIPK3 was assessed in the H/R and control groups. ^∗^*P* < 0.05 and ^∗∗^*P* < 0.01 vs. Control. The experiments were repeated at least three times. The results were expressed as mean ± SD.

**Figure 2:** Knockdown of circHIPK3 alleviates the kidney injury *in vitro*. (a) The transfection effectiveness was detected via qRT-PCR. *n* = 5. (b) Cell viability was measured in different groups. (c) The level of IL-1*β*, IL-6, and TNF-*α* was detected via ELISA. (d) The level of apoptosis-associated protein (Bcl2, Bax, and Cyt-c) was measured via western blot. (e) The production of ROS was evaluated. (f) The content of ATP was measured via the ATP Assay Kit. ^∗^*P* < 0.05 and ^∗∗^*P* < 0.01 vs. Control group and ^#^*P* < 0.05 vs. H/R group. The experiments were repeated at least three times. The results were expressed as mean ± SD.

**Figure 3:** circHIPK3 interacting with miR-93-5p regulates AKI progression. (a) Schematic diagram of bioinformatics prediction binding sites (upper). Luciferase assay report for circHIPK3 and miR-93-5p (lower). (b, c) The level of miR-93-5p was measured *in vivo* and *in vitro*. (d) The level of circHIPK3 and miR-93-5p was detected via qRT-PCR. (e) Cell viability was measured in different groups. (f) The level of IL-1*β*, IL-6, and TNF-*α* was detected via ELISA. (g) The production of ROS was evaluated. (h) The content of ATP was measured via ATP Assay Kit. (i) The apoptosis rate of the HK-2 cell after different treatments was detected via flow cytometry. ^∗^*P* < 0.05 vs. Control group, ^#^*P* < 0.05 vs. H/R group, and ^&^*P* < 0.05 vs. H/R+circHIPK3 group. The experiments were repeated at least three times. The results were expressed as mean ± SD.

**Figure 4:** KLF9 is a target of miR-93-5p. (a) Schematic diagram of bioinformatics prediction binding sites (upper). Luciferase assay report for KLF9 and miR-93-5p (lower). (b, c) The mRNA level of KLF9 was measured *in vivo* and *in vitro*. (d, e) The protein level of KLF9 was measured *in vivo* and *in vitro*. (f) The level of miR-93-5p and KLF9 was detected via qRT-PCR. (g) Cell viability was measured in different groups. (h) The production of ROS was evaluated. (i) The content of ATP was measured via ATP Assay Kit. (j) The apoptosis rate of HK-2 cell after different treatments was detected via flow cytometry. ^∗^*P* < 0.05 and ^∗∗^*P* < 0.01 vs. Control group, ^#^*P* < 0.05 vs. H/R group, ^&^*P* < 0.05 vs. H/R+KLF9 group, and ^&^*P* < 0.05 vs. H/R+KLF9 group. The experiments were repeated at least three times. The results were expressed as mean ± SD.

**Figure 5:** circHIPK3 is implicated in AKI via regulating the miR-93-5p/KLF9 axis. (a) AAV9 vector plasmid was injected into mice before operation. The level of circHIPK3, miR-93-5p, and KLF9 was detected via qRT-PCR. (b) The level of serum CREA, BUN, and uric acid in different groups. (c) Representative H&E images are shown in different groups. The section shows acute tubular necrosis characterized by loss of tubular epithelial cells. (d) Representative TUNEL staining images are shown in different groups. (e) The level of IL-1*β*, IL-6, and TNF-*α* was detected via ELISA. (f) The level of apoptosis-associated proteins (Bcl2, Bax, and Cyt-c) was measured via western blot. ^∗^*P* < 0.05 and ^∗∗^*P* < 0.01 vs. Sham group, ^#^*P* < 0.05 vs. I/R group, and ^&^*P* < 0.05 vs. I/R+circHIPK3 group. The experiments were repeated at least three times. The results were expressed as mean ± SD.

**Table 1:** Primers used in the qRT-PCR analysis.

Gene	Forward (5′-3′)	Reverse (5′-3′)
*circHIPK3*	TTCAACATGTCTACAATCTCGGT	ACCATTCACATAGGTCCGT
*miR-93-5p*	ACCATTCACATAGGTCCGTGAGCTGCCC	CTCAACTGGTGTCGTGGA
*Klf9*	CGAGCGGCTGCGACTACCTG	GGGCTGTGGGAAGGACTCGAC
*U6*	GCTTCGGCAGCACATATACT	GTGCAGGGTCCGAGGTATTC
*Gapdh*	AGGTCGGTGTGAACGGATTTG	TGTAGACCATGTAGTTGAGGTCA

## Data Availability

All data, models, and code generated or used during the study appear in the submitted article.
